RETRACTED

# The impact of seed burial depths and post-emergence herbicides on seedling emergence and biomass production of wild oat (*Avena fatua* L.): Implications for management

**DOI:** 10.1371/journal.pone.0240944

**Published:** 2020-10-28

**Authors:** Muhammad Mudassar Maqbool, Shazia Naz, Tasneem Ahmad, Muhammad Shahid Nisar, Hassan Mehmood, Mona S. Alwahibi, Jawaher Alkahtani

**Affiliations:** 1 Department of Agronomy, Faculty of Agricultural Sciences, Ghazi University, Dera Ghazi Khan, Pakistan; 2 Pakki Thatti Research & Development Farm, Toba Tek Singh, Pakistan; 3 Department of Plant Protection, Faculty of Agricultural Sciences, Ghazi University, Dera Ghazi Khan, Pakistan; 4 Department of Soil Science, Bahauddin Zakariya University, Multan, Pakistan; 5 Department of Botany and Microbiology, College of Science, King Saud University, Riyadh, Saudi Arabia; Harran University, TURKEY

## Abstract

Wheat (*Triticum aestivum* L) is among the most important cereal crops widely cultivated in the world. Wild oat (*Avena fatua* L.) competes with wheat for moisture, sunlight, space and nutrition. The successful management of weeds requires sound knowledge of their biology and response to different herbicides. This study inferred the impact of different constant temperature regimes and seed burial depths on seedling emergence and biomass production of wild oat. Moreover, the impact of different post-emergence herbicides applied at different growth stages on biomass production of wild oat was tested. The influence of different wild oat-wheat density (WWD) combinations on biomass production of wheat and wild oat was also inferred. Different constant temperature regimes significantly altered seed germination and biomass production of wild oat. The highest seed germination percentage and biomass production were noted under 15°C and 20°C, whereas the lowest values were recorded under 30°C. Similarly, days to start emergence, seedling emergence percentage and biomass production of wild oat was significantly affected by different seed burial depths. The lowest and the highest values of these parameters were observed under 4 and 10 cm depth, respectively. Different post-emergence herbicides and wild oat growth stages significantly altered biomass production. The highest reduction in fresh and dry biomass was recorded with herbicides’ application at 2–4 leaf stage compared with anthesis stage. Clodinofop resulted in higher reduction of fresh biomass, whereas higher reduction in dry biomass was noted with Sulfosulfuron. Seed germination of both species was not affected by different WWD combinations, except for the treatment where no seed was sown of both species. These results indicate that deep burial of seeds could prevent seedling emergence, whereas post-emergence herbicides must be applied at 2–4 leaf stage of wild oat for its effective management.

RETRACTED

## Introduction

Wheat (*Triticum aestivum* L.) gives life to one third of the global population, which consume it as staple food [1]. It is used as staple diet in various countries of the world; thus, ranked among the most important grain crops [2]. Wheat is extensively grown in the world as it was cultivated on 237 million hectares, with 25.19 million tons grain production during 2017–2018 [3]. Wheat occupies a dominant place in agricultural policies [2] and significantly contributes towards gross domestic product and value added in agriculture [2]. The average yield of wheat crop is much lower than its yield potential in many countries of the world [3]. Several biotic and abiotic constraints are responsible for low wheat yield in these countries. Weed infestation causes significant yield reduction, which may reach ~40%. The yield reduction caused due to weed infestation in wheat incurs billions of losses in the world [4].

Weed infestation significantly alters morphological and physiological characteristics of crop plants, which result in significant yield losses [5–7]. The duration and intensity of weed infestation affect the losses caused to crop production. Increasing duration of weed-crop competition poses negative impacts on yield-related attributes of different crops [8–10]. The density of the infesting weeds should be kept below economic threshold level during the critical period of competition [11–13]. Weeds compete with crop plants for resources and this competition significantly reduces yield [7, 9, 14]. The crop yields are reduced by ~50% due to weed infestation under certain circumstances [15]. Therefore, weed management is necessary in field crops to avoid economic losses.

Wild oat (*Avena fatua* L.) is a noxious weed, infesting wheat crop in rainfed and irrigated areas of the world [16–20]. Wild oat causes 20–76% yield losses in wheat crop depending upon the severity and duration of infestation. Different studies have reported that wild oat severely hampers yield components of wheat crop in different regions of the world [11, 21–24]. High temperature reduces seed viability and seed germination percentage of wild oat [25]. Low temperature did not affect the seed viability, although it is a species of semi-arid climates. Moreover, low seed germination under high temperature recruits lower number of seedlings, which ultimately reduces dry biomass production. Integrated weed management practices, including mechanical, chemical and biological methods are recommended for field crops [26–29].

RETRACTED

Manual weeding minimizes weed density; however, it incurs heavy labor costs and cannot be useful for farmers. On the other hand, mechanical methods are costly due to high fuel consumption and price [30]. Weed control with herbicides is quite effective and cheaper than the rest of the weed control methods [31–33]. However, increasing environmental and human health concerns on herbicides are being discussed in the recent era [34, 35]. Post emergence herbicides are an effective tool to lower weed-crop competition. Several herbicides are available, which can control wild oat [36, 37]. The herbicides are becoming ineffective due to the evolution of herbicide resistance [38]. Numerous studies have reported that herbicides application lowered weed infestation and increased wheat yield [4, 36].

Proper and effective management of wild oat is essential as it severely competes with wheat plants after its emergence. Successful management of any weed species requires sound knowledge of species’ biology, ecology, germination and emergence patterns and response to applied herbicides. Therefore, current study was designed to explore the impact of different constant temperature regimes and seed burial depths on seed germination and seedling emergence of wild oat. The second aim of the study was to explore the effect of different post emergence herbicides and WWD combinations on biomass production of wild oat. The results of the study will contribute towards the development of effective management strategies against wild oat.

## Materials and methods

One laboratory and three greenhouse experiments were performed to infer the impact of constant temperature regimes, seed burial depths, post emergence herbicides and WWD combinations on seed germination and seedling emergence and biomass production of wild oat.

### Seed collection

Wild oat seeds were collected from the wheat field in Dera Ghazi Khan. The seeds were stored at room temperature and used in the experiments. The seeds of wheat cultivar Ujala were collected from Ayub Agriculture Research Institute, Faislabad. The seed collection required no permission and did not involve any endangered species.

### Experiment 1: Effect of different constant temperature regimes on seed germination of wild oat

Seed germination of wild oat was recorded under five different constant temperature regimes (i.e., 10, 15, 20, 25 and 30°C). The experiment was conducted in automated incubators under laboratory conditions. The germination was assessed in Petri dishes (90 × 15 mm), having two layers of Whatman No. 1 filter paper. Deionized water was used to provide the required moisture to the seeds. Two Petri dishes were considered as one replication and 25 seeds were placed in each Petri dish. All temperature regimes were replicated four times. Incubators were adjusted at the desired temperatures and seeds were incubated. Germination was evaluated 21 days after experiment initiation [39, 40].

RETRACTED

### Experiment 2: Effect of seed burial depths on seedling emergence of wild oat

Seedling emergence of wild oat was recorded from four different seed burial depths (i.e., 4, 6, 8 and 10 cm) to infer the seed burial depth required for ceasing seedling emergence. The experiment was conducted in pots. The same sized seeds of wild oat were sown in the pots at the prescribed burial depths. The seeds were placed at equal distance in the pots to ensure that the seeds not face any competition in germination. Free draining, 8.8 liter pots were used in the study, which were filled with 2.7 kg of soil [41].

### Experiment 3: Effect of different wild oat-wheat densities on the growth of each other

Five different wild oat-wheat density (WWD) combinations were evaluated for their impact on seed germination and biomass production of both species. Seeding density of both species was kept inversely proportional to each other in WWD combinations. The WWD combinations were 0:8, 2:6, 4:4, 6:2 and 0:8 (wild oat:wheat). Free draining, 8.8 liter pots were used in the study. The pots were filled with 2.7 kg of soil and then seedlings were transplanted.

### Experiment 4: Effect of post-emergence herbicides on biomass production of wild oat

Efficacy of two post-emergence herbicides on biomass production of wild oat was tested. The experiment included two different factors, i.e., post-emergence herbicides and growth stages of wild oat. Two different post-emergence herbicides, i.e., Clodinofop and Sulfosulfuron at recommended doses (400 g ha^-1^ for Clodinofop and 35 g ha^-1^ for Sulfosulfuron) were tested, while distilled water was applied in the control treatment. These herbicides were applied at two different growth stages, i.e., 2–4 leaf and anthesis stage of wild oat.

### Experimental setup and design

The experiments 1–3 were conducted according to completely randomized design with four replications. The experiment 4 was conducted according to randomized complete block design with split plot arrangements. Post-emergence herbicides were kept in main plot, while growth stages of wild oat were regarded as sub-plots. All experiments were repeated over time (two experimental runs for each experiment).

### Data collection

Seed germination (experiment 1 and 3) and seedling emergence (experiment 2) was recorded daily and terminated 21 days after the start of experiments. Visible appearance of the cotyledon was taken as criterion for seed germination and seedling emergence. The day at which first seedling emerged was considered as days to start emergence. The percentage of the emerged seedlings was computed using the following equation;

$$Seedling\;emergence\;(\%)=\frac{Total\;number\;of\;seedlings\;emerged}{Total\;number\;of\;seeds\;sown}\times 100$$

All seedlings were taken off from the pots at the termination of experiments, divided into shoots and roots, weighed fresh and dried in an oven at 70°C for 72 hours. The dried roots and shoots were weighed to record root and shoot dry weight pot^-1^.

RETRACTED

### Statistical analysis

The data of all experiments were analyzed and interpreted separately. The differences among experimental runs were tested by paired *t* test, which were non-significant. Therefore, data of both experimental runs were pooled. The collected data were subjected to Fisher’s Analysis of Variance (ANOVA) (one-way for experiment 1, 2 and 4 and 2-way for experiment 3) technique [42]. The normality in the data was tested prior to ANOVA by Shapiro-Wilk normality test [43] and parameters showing non-normal distribution were transformed using arcsine transformation techniques to meet the normality assumption. The treatment means were compared by least significant difference test at 95% probability level where ANOVA indicated significance. The ANOVA was performed on SPSS version 21.0 [44].

## Results

### Experiment 1: Effect of different constant temperature regimes on seed germination of wild oat

Different constant temperature regimes significantly altered days to start emergence (DE), seed germination percentage (G%) and fresh and dry biomass of wild oat (Table 1). The DE were initially reduced with increasing temperature and then an increase was recorded. The lowest number of DE were taken by the seeds incubated under 15°C and 20°C, whereas the highest DE were taken by the seeds incubated at 30°C (Fig 1A).

**Fig 1:** The effect of different constant temperature regimes on days to start emergence (A), seed germination percentage (B), seedling fresh weight (C) and seedling dry weight (D) of wild oat.

**Table 1:** Analysis of variance for days to start emergence, seed germination percentage and seedling fresh and dry biomass of wild oat under different constant temperature regimes.

Source	DF	Sum of squares	Mean squares	F value	P value
**Days to start emergence**					
**Temperature regimes**	4	19.30	4.82	28.95	0.0000*
**Error**	15	2.50	0.16		
**Total**	19	21.80			
**Seed germination percentage**					
**Temperature regimes**	4	2482.50	620.62	67.70	0.0000*
**Error**	15	137.50	9.16		
**Total**	19	2620.00			
**Seedling fresh weight**					
**Temperature regimes**	4	147.70	36.92	146.24	0.0000*
**Error**	15	3.78	0.25		
**Total**	19	151.49			
**Seedling dry weight**					
**Temperature regimes**	4	40.28	10.07	235.93	0.0000*
**Error**	15	0.64	0.04		
**Total**	19	40.92			

DF = degree of freedom

* = significant

The G% was increased with increasing temperature up to 20°C and then declined. The highest G% was noted under 15°C and 20°C, while the lowest was recorded under 10°C and 30°C (Fig 1B). Seedling fresh weight was increased with increasing temperature until 20°C and then a constant reduction was noted. The highest and the lowest seedling fresh weight was noted under 20°C and 30°C, respectively (Fig 1C). Seedling dry weight increased with increasing temperature until 20°C and then a constant reduction was noted. The highest and the lowest seedling dry weight was noted under 20°C and 30°C, respectively (Fig 1D).

RETRACTED

### Experiment 2: Effect of seed burial depths on seedling emergence of wild oat

Different seed burial depths significantly altered DE, final emergence percentage (FEP) and fresh and dry biomass production of roots and shoots (Table 2). Increasing seed burial depth increased DE. The highest number of DE (10.50) were taken under 10 cm seed burial depth, whereas the lowest (4.25) DE was recorded for 4 cm burial depth (Fig 2A). The FEP was linearly deceased with increasing seed burial depth. The highest FEP (87.75%) was recorded under shallow depth, i.e., 4 cm, whereas the lowest FEP (20.00%) was recorded for the deepest seed burial treatment, i.e., 10 cm (Fig 2B).

**Fig 2:** The effect of different seed burial depths on days to start emergence (A), seedling emergence percentage (B), shoot fresh weight (C), shoot dry weight (D), root fresh weight (E) and root dry weight (F) of wild oat.

**Table 2:** Analysis of variance for days to start emergence, root and shoot fresh and dry biomasses of wild oat under different seed burial depths.

Source	DF	Sum of squares	Mean squares	F value	P value
**Days to start emergence**					
**Seed burial depths**	3	86.50	28.83	98.86	0.0000*
**Error**	12	3.50	0.29		
**Total**	15	90.00			
**Seedling emergence percentage**					
**Seed burial depths**	3	9993.50	3331.17	1095.18	0.0000*
**Error**	12	36.50	3.04		
**Total**	15	10030.00			
**Shoot fresh weight**					
**Seed burial depths**	3	682.38	227.46	757.74	0.0000*
**Error**	12	3.60	0.30		
**Total**	15	685.98			
**Shoot dry weight**					
**Seed burial depths**	3	73.80	24.60	187.82	0.0000*
**Error**	12	1.57	0.13		
**Total**	15	75.37			
**Root fresh weight**					
**Seed burial depths**	3	118.60	39.60	455.41	0.0000*
**Error**	12	1.07	0.08		
**Total**	15	119.85			
**Root dry weight**					
**Seed burial depths**	3	21.39	7.13	59.37	0.0000*
**Error**	12	1.44	0.12		
**Total**	15	22.83			

DF = degree of freedom

* = significant

The highest fresh shoot biomass (25.07 g pot^-1^) was recorded under 4 cm seed burial depth, whereas the lowest (7.74 g pot^-1^) was noted under 10 cm (Fig 2C). Dry shoot biomass production linearly decreased with increasing seed burial depth. The highest dry shoot biomass (9.63 g pot^-1^) was recorded under 4 cm, whereas the lowest (3.77 g pot^-1^) was observed under 10 cm seed burial depth (Fig 2D).

RETRACTED

Fresh root biomass production linearly decreased with increasing seed burial depth. The highest fresh root biomass (11.47 g pot^-1^) was recorded under 4 cm seed burial depth, whereas the lowest (4.17 g pot^-1^) was noted under 10 cm seed burial depth (Fig 2E). Dry root biomass production linearly decreased with increasing seed burial depth. The highest dry root biomass (5.63 g pot^-1^) was recorded under 4 cm seed burial depth, whereas the lowest (2.52 g pot^-1^) was observed under 10 cm seed burial depth (Fig 2F).

### Experiment 3: Effect of different wild oat-wheat densities on the growth of each other

Different wild oat-wheat density (WWD) combinations significantly altered seed germination and biomass production of both species and number of tillers per plant of wheat (Table 3). Seed germination of wheat remained same under all WWD combinations except 8:0 (Fig 3A).

**Fig 3:** The effect of different wild oat and wheat density combinations on seed germination (A), number of tillers per plant (B), fresh weight (C) and dry weight (D) of wheat.

**Table 3:** Analysis of variance for seed germination percentage and fresh and dry biomasses of wild oat and wheat and number of tillers per plant of wheat under different wild oat-wheat density combinations.

Source	DF	Sum of squares	Mean squares	F value	P value
**Seed germination percentage (wheat)**					
**Density combinations**	4	28169.40	7042.36	48.10	0.0000*
**Error**	15	2196.40	146.43		
**Total**	19	30365.80			
**Number of tillers per plant (wheat)**					
**Density combinations**	4	254.80	63.70	123.29	0.0000*
**Error**	15	7.75	0.51		
**Total**	19	262.55			
**Fresh weight (wheat)**					
**Density combinations**	4	42287.40	10571.80	1559.61	0.0000*
**Error**	15	101.70	6.80		
**Total**	19	42389.10			
**Dry weight (wheat)**					
**Density combinations**	4	4311.97	1077.99	1169.29	0.0000*
**Error**	15	13.83	0.92		
**Total**	19	4325.80			
**Seed germination percentage (wild oat)**					
**Density combinations**	4	27588.40	6897.09	32.64	0.0000*
**Error**	15	3169.50	211.30		
**Total**	19	30757.90			
**Fresh weight (wild oat)**					
**Density combinations**	4	26966.70	6741.69	2931.04	0.0000*
**Error**	15	34.50	2.30		
**Total**	19	27001.20			
**Dry weight (wild oat)**					
**Density combinations**	4	4276.73	1069.18	1693.65	0.0000*
**Error**	15	9.47	0.63		
**Total**	19	4286.20			

DF = degree of freedom

* = significant

Fresh and dry biomass production of wheat decreased with increasing wild oat density and decreasing wheat density. The highest fresh and dry biomass production of wheat were recorded under 0:8 (0 wild oat seeds and 8 wheat seeds), whereas the lowest fresh and dry biomass production were recorded for 8:0 (Fig 3C and 3D). Number of tillers per plant decreased with increasing wild oat density and decreasing wheat density. The highest number of tillers per plant was recorded under 0:8, whereas the lowest was recorded for 8:0 (Fig 3B).

RETRACTED

Seed germination of wild oat remained same under all density combinations except 0:8 (0 seeds per pot of wild oat and 8 seeds of wheat). These results indicated that different WWD combinations did not affect the seed germination of wild oat (Fig 4A).

**Fig 4:** The effect of different wild oat and wheat density combinations on seed germination (A), fresh weight (B) and dry weight (C) of wild oat.

Fresh biomass of wild oat decreased with increasing wheat density and decreasing wild oat density. The highest fresh biomass was recorded under 8:0 (8 wild oat seeds and 0 wheat seeds), whereas the lowest was noted for 0:8 (Fig 4B). Dry biomass decreased with increasing wheat density and decreasing wild oat density. The highest dry biomass production was recorded under 8:0 (Fig 4C).

### Experiment 4: Effect of post emergence herbicides on biomass production of wild oat

Different growth stages of wild oat did not affect the fresh biomass production; however, it was significantly altered by different post-emergence herbicides and growth stages by post-emergence herbicides’ interactions (Table 4). Different post-emergence herbicides reduced fresh biomass and application at 2–4 leaf stage resulted in higher reduction of fresh biomass. The highest fresh biomass was observed at 2–4 leaf growth stage with control treatment of the study. The lowest fresh biomass was noted for Clodinofop applied at 2–4 leaf stge. Overall; Clodinofop better suppressed the fresh biomass compared to Sulfosulfuron (Fig 5A).

**Fig 5:** The effect of different post-emergence herbicides on fresh biomass (A) and dry biomass production (B) of wild oat.

**Table 4:** Analysis of variance for and fresh and dry biomass of wild oat under different post-emergence herbicides’ application.

Source	DF	Sum of squares	Mean squares	F value	P value
**Fresh biomass**					
**Growth Stage (G)**	1	4.62	4.62	8.31	0.06^NS^
**Herbicides (H)**	2	229.04	114.52	131.13	0.000*
**G × H**	2	27.40	13.72	15.71	0.000*
**Dry biomass**					
**Growth Stage (G)**	1	27.26	27.26	75.35	0.003*
**Herbicides (H)**	2	158.01	79.00	785.79	0.000*
**G × H**	2	20.01	10.00	99.54	0.000*

DF = degree of freedom

* = significant

Different growth stages, post-emergence herbicides and growth stages by post-emergence herbicides’ interactions significantly altered dry biomass production of wild oat (Table 4). Herbicide application at 2–4 leaf stage resulted in higher reduction of dry biomass. The highest dry biomass was observed at 2–4 leaf growth stage with control treatment. The lowest dry biomass was noted for Sulfosulfuron applied at 2–4 leaf stage. Overall, Sulfosulfuron better suppressed dry biomass compared to Clodinofop (Fig 5B).

RETRACTED

## Discussion

Seed germination percentage is an important ecological trait defining the establishment success and failure of wild and cultivated plant species. Higher seed germination percentage ensures better plant population. Temperature is an imperative determinant of seed germination and different seeds germinate at a specific temperature range. Seed germination percentage determines the density of a species in field. Higher seed germination guarantees high density, whereas species having low seed germination end with low density. Numerous factors alter the seed germination of weed species. These factors include temperature, light, soil pH, osmotic potential, hormones and seed burial depth. Among these factors, temperature affects several hormones playing role in seed germination [39, 40, 45–48]. Different species, and even the populations of same species have specific temperature requirements for seed germination [49, 50].

Temperature is an important ecological factor affecting the seed germination by activating different enzymes [39, 40, 45–48]. High temperature reduces seed viability and germination percentage of wild oat [25]. Wild oat shows higher seed germination during spring compared to the autumn season [25]. Wild oat germinates under a wide range of temperature regimes (5–30°C). However, several studies have reported that the optimum temperature for the seed sprouting of wild oat is 15–20°C [25]. Like other species, wild oat has a specific soil temperature requirement for seed germination [51]. Seed germination of wild oat starts once the soil temperature is raised 4–8°C and continues until 17°C. Beyond this temperature, seed germination slows down and ultimately ceases with further increase in temperature. The low dry biomass under high temperature in the current study can be explained by the lower temperature requirement of wild oat seeds for germination. Moreover, the lesser number of germinated seeds produced lesser seedlings, which ultimately resulted in low dry biomass Hassanein et al. [52] indicated that wild oat exhibits highest seed germination under 20°C, while produced the highest seedling dry weight under 25°C.

RETRACTED

The optimum time to control wild oat is at 2–3 seedlings/m^2^ [53]. Different plant species exhibit differential requirements for optimum root growth mainly due to the nature of seeds and the environmental conditions faced by the seeds during seed germination [54]. Nonetheless, seedling emergence is hindered by lesser light diffusion in the deeper soil layers [55, 56], which results in poor root development. The viability of the seeds is increased when buried under shallow depth, whereas it is decreased when buried at deeper depths. The lesser light diffusion and reduced respiration are responsible for the reduced seed viability. It has been observed that seed viability and root growth of wild oat is decreased with increasing seed burial depth [57]. Therefore, the decreased root biomass with increasing seed burial depth is the collective result of less light diffusion, high mechanical impedance offered by the soil and decreased seed viability.

The cultural or mechanical weed control methods are less effective for wild oat compared to chemical control, which is the most effective for wild oat management [58, 59]. The urea family and phenoxypropionates herbicides are considered the most effective chemical control of wild oat. An extensive review has suggested that numerous herbicides are effective in controlling wild oat compared to the other methods [60]. These herbicides are effective when applied alone or in combination with other herbicides or adjuvants. Different herbicides which can effectively control wild oat are; atrazine, benzoylprop-ethyl, chlorsulfuron, chlorotoluron, clodinafop, cycloxydim, diclofop-methyl, difenzoquat, diflufenican, dimethenamid + trifluralin, fenoxaprop-ethyl and flamprop-isopropyl [25]. The higher reduction in fresh weight at 2–4 leaf growth stage indicated that wild oat gives better response to applied herbicides at initial stage compared to later stages.

The density of weeds and crop plants significantly affect the seed germination and growth traits of both species. The higher seed density of weed species negatively affect the seed germination and subsequent growth of crop plants. Moreover, higher seed density results in higher weed density in crop plants, which exerts serious negative impacts on crop yield. Seed germination of wheat was affected by increasing WWD and vice versa. This reduction in seed germination is the result of increase weed-crop competition, which reduced the seed germination percentage. Moreover, this weed-crop competition is depicted in growth and development as well.

RETRACTED

## Conclusion

Seed germination of wild oat is stimulated when temperature reaches 10°C; therefore, management strategies should be started once the soil temperature reaches 10°C. Increasing seed burial depth suppresses the seedling emergence of wild oat; therefore, burying wild oat seeds >10 cm deep and subsequent shallow tillage along with the management of emerging seedlings could be a viable management option. Wild oat better responded to applied herbicides at 2–4 leaf stage compared to anthesis stage; therefore, herbicides must be applied at 2–4 leaf stage for effective management.
